The article "Expression of Dickkopf-1 and Twist2 in Cervical Squamous Cell Carcinoma and Their Correlation with Vasculogenic Mimicry" was retracted in 2023. Reasons: signs of a paper mill; suspected computer-generated content; unreliable results or conclusions; concerns about the data.

# Expression of Dickkopf-1 and Twist2 in Cervical Squamous Cell Carcinoma and Their Correlation with Vasculogenic Mimicry

**DOI:** 10.1155/2022/9288476

**Published:** 2022-03-16

**Authors:** Beibei Wang, Huihui Zhang, Li Wei, Yan Li

**Affiliations:** Department of Gynecological Oncology, The 1st Affiliated Hospital of Bengbu Medical College, Bengbu 233000, China

## Abstract

Wnt/*β*-catenin signaling, epithelial-mesenchymal transition (EMT), and vasculogenic mimicry (VM) all exert important effects in tumors. Dickkopf-1 (DKK1) is an antagonist of the Wnt/*β*-catenin, Twist homolog 2 (Twist2) is a key EMT transcription factor involved in cancer cell migration and invasion, and VM participates in the progression and metastasis of a variety of cancers. However, the correlation of DKK1, Twist2, and VM in cervical squamous cell carcinoma(CSC) is still unclear. This study focuses on correlations among these factors as well as their correlation with clinicopathologic data and survival in CSC. DKK1, Twist2, and VM expressions were immunohistochemically examined in 116 CSC tissues and 37 normal cervical tissues. Furthermore, clinical data were processed. The expression levels of these three factors differed between CSC and normal tissues. VM was observed in CSC, but not in normal cervical tissues. Twist2 expression was high in CSC but low in normal cervical tissues, whereas DKK1 expression had the opposite pattern. Tumor cells with VM had a high expression of Twist2 and low expression of DKK1. In addition, DKK1 expression was negatively correlated with Twist2 expression. Analyzing the relationships of DKK1, Twist2, and VM with the data of patients with CSC revealed that DKK1 expression was negatively correlated with the clinical stage, degree of differentiation, depth of infiltration, and lymph node metastasis of tumors. VM and Twist2 expression were positively correlated with the degree of differentiation, the depth of infiltration, and lymph node metastasis. The positive rate of VM was greater in stage II than in stage I. The patients who expressed VM and Twist2 had a reduced overall survival (OS) when compared with patients not expressing these proteins. However, the patients who expressed DKK1 had an increased OS when compared with patients who did not show any DKK1 expression. Multivariate analysis indicated that the expressions of DKK1, Twist2, and VM were prognostic factors for CSC. VM and the expression of DKK1 and Twist2 can be the potential prognostic biomarkers and therapeutic targets for CSC.

## 1. Introduction

Cervical cancer is a common malignancy of the female reproductive system. The incidence in China is approximately 10.9 per 100,000 [1]. Although in recent years, treatment methods and techniques for cervical cancer have greatly improved, recurrence and metastasis are still the main reasons for treatment failure. Therefore, elucidating the mechanisms underlying cervical cancer invasion and metastasis is essential for intervention and control to improve the survival rate of cervical cancer patients.

The article "Expression of Dickkopf-1 and Twist2 in Cervical Squamous Cell Carcinoma and Their Correlation with Vasculogenic Mimicry" was retracted in 2023. Reasons: signs of a paper mill; suspected computer-generated content; unreliable results or conclusions; concerns about the data.

Solid tumors need blood supply for growth and new blood vessels will be formed to maintain this when the diameter of the tumor is more than 2 mm; otherwise, necrosis will occur due to ischemia and hypoxia [2]. The concept of vasculogenic mimicry (VM) was first proposed in 1999 by Maniotis et al. in a study of uveal melanoma in human eyes. VM is a pattern of tumor microcirculatory that differs from classical tumor angiogenesis because it does not rely on endothelial cells. VM is a reticular, duct-like structure that can transport blood (plasma, red blood cells). This structure is composed of tumor cells that have transformed themselves to mimic the blood vessels in the body. VM connects to the host blood vessel to provide the tumors with a blood supply, thereby remodeling the tumor microcirculation [3]. VM has the following characteristics: (1) there are no vascular endothelial cells on the inner wall of VM blood vessels; (2) tumor cells form vascular-like channels; (3) periodic acid Schiff (PAS) staining is positive and CD34 staining is negative, in contrast to the negative PAS staining and positive CD34 staining found in the endothelial vascular channel; and (4) plasma and RBCs are in the blood vessel-like channel [4, 5]. Because VM channels are composed of tumor cells and lack the barrier function of endothelial cells, they are more conducive to tumor invasion and metastasis. In addition, in terms of treatment, the discovery of VM has explained the ineffectiveness of anticancer drugs that target vascular endothelial cells alone. A series of studies have confirmed the existence of the VM phenomenon in a variety of malignant tumors, including osteosarcoma, liver, breast, colorectal, and prostate cancers, and its close relationships with tumor growth, invasion, metastasis, and prognosis [6–10]. Previous studies by our group also showed that VM exists in cervical squamous cell carcinoma (CSC) with poorer differentiation, higher clinical stage, or lymph node metastasis.

The tumor cells involved in the formation of VM lose the characteristics of epithelial cells and acquire the characteristics of endothelial cells. Endothelial cells are a type of mesenchymal cells. Thus, the differentiation of epithelial tumor cells into mesenchymal endothelial cells is likely to occur during VM formation, i.e., EMT. EMT is the process by which epithelial cells are transformed to mesenchymal cells via several steps, including reducing the expression of adhesion molecules, transforming the cytokeratin skeleton to the vimentin-based cytoskeleton, and acquiring the morphologies of mesenchymal cells [11]. EMT controls tumor cell formation by VM and promotes tumor invasion and metastasis through a variety of mechanisms. During this process, a series of changes occur in the expression of related marker proteins. For example, the epithelial markers E-cadherin, occludin-1, and *α*-catenin are gradually lost, whereas the mesenchymal markers VE-cadherin, fibronectin, and vimentin are upregulated; the downregulation of E-cadherin indicates EMT [12]. Many transcription factors that cause EMT during development, such as Slug [5], ZEB1 [10], ZEB2 [13], and Twist homolog 2 (Twist2) [14], can interact with the E-cadherin promoter to mediate transcriptional activity. E-cadherin is downregulated, cell adhesion ability is decreased, and cell invasion and metastasis are enhanced.

The article "Expression of Dickkopf-1 and Twist2 in Cervical Squamous Cell Carcinoma and Their Correlation with Vasculogenic Mimicry" was retracted in 2023. Reasons: signs of a paper mill; suspected computer-generated content; unreliable results or conclusions; concerns about the data.

Twist2 belongs to the class B basic helix-loop-helix protein (bHLH) family and regulates transcription in mesenchymal cell lineages during development. Twist2 directly binds the E-box consensus sequence in the gene-controlled region to achieve transcriptional regulation of target genes [15]. Twist2 is overexpressed in most tumors and contributes to occurrence and progression. The positive expression rate of Twist2 in glioma is 90% (54/60) vs. 30% (6/20) in nontumor brain tissues, and its level is positively correlated with the malignant grade of glioma. Twist2 may regulate tumor metastasis through EMT [14], but there have been few studies of Twist2 in CSC.

The canonical Wnt/*β*-catenin signaling pathway is one of the most important signaling pathways in human malignancies, as it is involved in cell proliferation, differentiation, and angiogenesis. The Wnt signaling pathway is inhibited by many different antagonistic molecules, and five such groups of molecules have been identified so far: secreted frizzled-related proteins (sFRPs), Wnt inhibitory factory-1 (WIF-1), Xenopus Cerberus, Wise, and the Dickkopf (DKK) secretory protein family [16]. The DKK gene family is a small, evolutionarily conserved gene family that includes DKK1, DKK2, DKK3, DKK4, and soggy [17]. The most studied member is DKK1, a secreted protein that binds lipoprotein receptor-related proteins 5 and 6 (LRP5/6). It blocks Wnt-1 signaling and acts as a general inhibitor of the Wnt signaling pathway. DKK1 has antitumor effects in colon cancer, breast cancer, and cervical cancer [18–20].

The Wnt/*β*-catenin signaling pathway, EMT, and VM are all important processes of malignant tumor invasion and metastasis. This study examined the expression of the Wnt/*β*-catenin signaling pathway regulatory protein DKK1, the EMT marker protein Twist2, and VM in CSC and normal cervical tissues, as well as their relationships with clinicopathological factors. The relationships among the Wnt/*β*-catenin signaling pathway, EMT, and VM were preliminarily analyzed to provide an experimental basis for the study of new targets and drugs to combat tumor angiogenesis.

The article "Expression of Dickkopf-1 and Twist2 in Cervical Squamous Cell Carcinoma and Their Correlation with Vasculogenic Mimicry" was retracted in 2023. Reasons: signs of a paper mill; suspected computer-generated content; unreliable results or conclusions; concerns about the data.

In this study, the expression of DKK1 Twist2, and VM in normal cervical and CSC tissues was detected by immunohistochemistry. In addition, the relationships between protein expression and the pathologic findings of CSC and between protein expression and prognoses were further analyzed to provide a clinical basis for cervical cancer.

## 2. Proposed Method

We retrospectively collected 116 CSC tissue specimens that were filed and embedded in the Department of Clinical Pathology, the First Affiliated Hospital of Bengbu Medical College, China, from January 2014 to December 2015 with approval by the 1st Affiliated Hospital of Bengbu Medical College and followed relevant guidelines and regulations. There was no preoperative radiotherapy, chemotherapy, or other antitumor treatment and no other combined tumor types among these patients. All patients had complete clinical data. Another 37 normal cervical tissues resected due to uterine fibroids within the same time frame were selected and confirmed as normal by pathological HE staining. The average age was 45 years (range: 25–78 years). 40 patients were <45 years old and 76 were ≥45 years old. The pathological grades included 31 cases of high differentiation, 68 cases of moderate differentiation, and 17 cases of poor differentiation. There were 47 cases with infiltration depth <1/2, 69 cases with infiltration depth ≥1/2, 51 cases with tumor diameter <4 cm, and 65 cases with tumor diameter ≥4 cm. According to the International Federation of Gynecology and Obstetrics (FIGO) staging (2009), there were 75 cases of stage I and 41 cases of stage II. There were 35 cases of lymph node metastasis and 81 cases of non-metastasis.

DKK1 rabbit polyclonal antibody, TWIST2 mouse monoclonal antibody, and CD34 rabbit monoclonal antibody were all purchased from Proteintech Group, Inc. The max vision kit and DAB color development kit were provided by Fuzhou Maixin Biological Company.

Specimens were fixed, embedded, and sectioned with a thickness of 4 *μ*m. The slices were baked, deparaffinized in xylene solution, and dehydrated in graded ethanol solution. All procedures were carried out according to the manual of the kit. Known positive slices were used as controls, and PBS solution was used instead of the primary antibody as a blank control.

The article "Expression of Dickkopf-1 and Twist2 in Cervical Squamous Cell Carcinoma and Their Correlation with Vasculogenic Mimicry" was retracted in 2023. Reasons: signs of a paper mill; suspected computer-generated content; unreliable results or conclusions; concerns about the data.

Specimens were stained with CD34. After 3,3′-diaminobenzidine color development, the specimens were rinsed with running water for 1 min to terminate the color development reaction and then oxidized in 0.5% periodic acid for 10 min. After washing with running water for 2 min, the samples were immersed in the Schiff solution and stained for 15–30 min, rinsed with distilled water 3 × 1 min, rinsed with distilled water for 3–5 min, lightly stained with hematoxylin to visualize nuclei, fractionated in alcohol with hydrochloric acid, returned to blue, dehydrated, transparentized, and sealed into slides with a neutral gum.

The positive expression of DKK1 was defined as a mainly cytoplasmic expression with occasional expression in the nucleus; cells with brown-yellow granules in the cytoplasm were considered positive. A Twist2-positive signal was dark brown and localized in the cytoplasm and/or nucleus. The determination was made by the secondary scoring method of dye intensity and color range. Scoring based on the percentage of positive cells was as follows: less than 10%, 0 points, 10–25%, 1 point, 26–50%, 2 points; and more than 50%, 3 points. Staining intensities of colorless, light yellow, brown-yellow, and dark brown were recorded as 0, 1, 2, and 3 points, respectively. The two scores were multiplied; a positive expression index >3 was defined as positive immunohistochemical staining and ≤3 was defined as negative staining.

The existence of VM was verified by CD34/PAS dual staining. Under a microscope, CD34-positive granules were expressed in the plasma of vascular endothelial cells and stained as brown color. PAS-positive expression was observed in the basement membrane of vascular or vascular-like luminal walls, with a purplish or cherry-red color. VM was a vascular-like structure surrounded by deformed CSC cells, without CD34 staining, but lined with a basement membrane-like structure surrounded by a layer of PAS-positive material. Red blood cells could be seen inside, and there was no surrounding bleeding, necrosis, or inflammatory cell infiltration. The immunohistochemistry and CD34/PAS dual staining results were checked by two pathologists.

Data were processed with SPSS 20.0 software. The differential expression of DKK1, Twist2, and VM in CSC and normal cervical tissues, as well as their association with various clinicopathological parameters, was statistically analyzed with the Fisher exact test or Chi-square test. In addition, a Kaplan–Meier survival curve was used to evaluate the survival analysis, a log-rank test was used to compare survival rates, and Cox regression analysis was used to analyze prognostic factors. *P* < 0.05 was considered statistically significant.

The article "Expression of Dickkopf-1 and Twist2 in Cervical Squamous Cell Carcinoma and Their Correlation with Vasculogenic Mimicry" was retracted in 2023. Reasons: signs of a paper mill; suspected computer-generated content; unreliable results or conclusions; concerns about the data.

## 3. Analysis and Results

### 3.1. DKK1, Twist2, and VM Expression in CSC and Normal Cervical Tissues

The *χ*2 test exhibited that the expression of DKK1 was lower in CSC than in normal cervical tissues (44.8% vs. 67.6%) (*P* < 0.05), as shown in Figures 1(a) and 1(b). The expression of Twist2 was higher in CSC than in normal cervical tissues (69.0% vs. 37.8%, *P* < 0.01), as shown in Figures 1(c) and 1(d). The VM-positive detection rate in CSC was 23.3% (27/116), whereas there was no presence of VM in normal cervical tissues (*P* < 0.01), as shown in Figures 1(e) and 1(f).  Table 1 displays the expression of DKK1, Twist2, and VM in CSC and normal cervical tissues.

### 3.2. Expression of DKK1, Twist2, and VM in CSC and their Association with Clinicopathological Parameters

The positive expression rate of the DKK1 protein in CSC was associated with tissue differentiation, depth of infiltration, clinical stage, and lymph node metastasis. The poorer the differentiation, the deeper the infiltration, and the higher the clinical stage, the lower the positive expression rate of the DKK1 protein (*P* < 0.05). The positive expression rate of DKK1 was lower in the lymph node metastasis group than the nonmetastatic group (*P* < 0.01). Twist2 was positively expressed in CSC more often than in normal tissues. With poorer differentiation, deeper infiltration, and lymph node metastases, the positive rate of Twist2 was higher (*P* < 0.05). Positive VM expression was positively correlated with the clinical stage, histological grade, depth of infiltration, and lymph node metastasis. The data are shown in Table 2.

### 3.3. Differences in DKK1 Expression between the VM+ and VM–Groups in the CSC

In the VM-negative group, 45 cases (50.6%, 45/89) were positive for DKK1 expression, whereas 7 cases (25.9%, 7/27) in the VM-positive group were positive for expression of DKK1. The difference in DKK1 expression between the VM-positive and VM-negative groups was significant (*P* < 0.05). DKK1 expression was absent in the VM-positive group.  Table 3 displays the relationship between VM and DKK1.

### 3.4. Differences in the Expression of Twist2 between the VM+ and VM–Groups in CSC

Twist2 was highly expressed in the VM-positive group. Of the 89 tissues in the VM-negative group, Twist2 expression was positive in 57cases (64.0%) whereas, among the 27 tissues in the VM-positive group, Twist2 expression was positive in 23 cases (85.2%). The difference between the two groups was significant (*P* < 0.05).  Table 4 illustrates the relationship between VM and Twist2.

The article "Expression of Dickkopf-1 and Twist2 in Cervical Squamous Cell Carcinoma and Their Correlation with Vasculogenic Mimicry" was retracted in 2023. Reasons: signs of a paper mill; suspected computer-generated content; unreliable results or conclusions; concerns about the data.

### 3.5. Correlation between Twist2 and DKK1 Protein Expressions in CSC

Among the 116 cervical cancer tissues, 80 were positive for Twist2 expression, among which 30 cases (37.5%) were also positive for DKK1 expression. In the remaining 36 cases, Twist2 expression was negative and 22 of these were positive for DKK1 expression (61.1%). The difference between DKK1 and Twist2 expression was significant (*P* < 0.05). The DKK1 expression rate was lower in the Twist2-positive group.  Table 5 shows the relationship between DKK1 and Twist2.

## 4. Survival Analysis

Follow-up data suggested that the clinical stage, metastasis, and the expression of DKK1, Twist2, and VM had significant effects on the survival rate of patients (*P* < 0.05); the Kaplan–Meier analysis revealed that the OS time of the subjects who expressed Twist2 and VM was lower than the patients without expressions (*P*=0.008, *P*=0.001); the OS time of the patients who expressed DKK1 was higher than the subjects without expression (*P*=0.005); the OS of patients with lymph node metastasis, stage III lower than those without lymph node metastasis, stage II. The multivariate analysis suggests that DKK1, Twist2, and VM are independent prognostic indicators for CSC.  Table 6 shows results of univariate analyses of overall survival (OS) time.  Table 7 presents Cox multivariate analysis of the three factors and patient mortality.  Figure 2 shows the Kaplan–Meier analysis of the survival rate of patients with CSC.

Tumor occurrence, progression, invasion, and metastasis depend on tumor angiogenesis. VM is a newly described microcirculatory pattern that differs from classical tumor angiogenesis because it can provide a sufficient blood supply which does not rely on endothelial cells. VM greatly limits the therapeutic efficacy of antiangiogenic drugs. Although in-depth studies have made great progress in understanding VM, the mechanism underlying VM formation has not yet been fully elucidated. Because the concept of VM was proposed in 1999, many studies have confirmed that VM exists in a variety of malignant tumors and suggested that VM indicates a poor prognosis.

Compared with these previous studies, the current study included more cases. Among 116 included CSCs, 27 (23.3%) had VM, while VM was absent in all normal cervical tissues (*P* < 0.05). VM expression in CSC was closely correlated with the FIGO stage, degree of differentiation, depth of infiltration, and presence of lymph node metastasis (*P* < 0.05). The OS time of CSC patients who expressed VM was lower than the subjects without expression. We conclude that VM should be considered a usefully prognostic biomarker for CSC. Possibly because VM channels consist of only one layer of the basement membrane and relatively loosely connected tumor cells and thus lack the barrier function of endothelial cells, making it easier for tumor cells to enter the blood circulation and metastasize. During the transformation of tumor cells into VM, EMT plays a key role in promoting tumor invasion and metastasis through a variety of mechanisms, including the upregulation of EMT transcription factors such as Snail and Twist, as well as matrix metalloproteinase 2. Twist2 is an indicator of cervical cancer metastatic potential. A high expression of Twist2 enhances cell migration ability and promotes EMT.

The article "Expression of Dickkopf-1 and Twist2 in Cervical Squamous Cell Carcinoma and Their Correlation with Vasculogenic Mimicry" was retracted in 2023. Reasons: signs of a paper mill; suspected computer-generated content; unreliable results or conclusions; concerns about the data.

We used immunohistochemistry to preliminarily analyze the expression of Twist2 in CSC and their differential expression between the VM-positive and VM-negative groups. The results showed that Twist2 was positively expressed in tumor cells more often than in normal cells and that it was mainly expressed in tumor tissues with a low degree of differentiation, deep infiltration depth, or lymph node metastasis. Twist2 expression was different between the tumor tissues and control tissues (*P* < 0.05). Twist2 was expressed in 23/27 cases in the VM-positive group (85.2%), a greater frequency than in the VM-negative group (*P* < 0.05). We hypothesize that Twist2 expression promotes tumor invasion and metastasis. Furthermore, the OS analysis indicated that the patients who expressed Twist2 survived shorter than those without expression. We conclude that Twist2 should be considered a usefully prognostic biomarker for CSC. The Wnt signaling pathway is an evolutionarily conserved signaling pathway that is critical for many biological activities, including embryonic development, cell growth, migration, differentiation, and normal tissue reconstruction. The Wnt pathway is turned off in normal mature cells. Overactivation or dysregulation of the Wnt signaling pathway will lead to an abnormal body development, tumor formation, or other diseases. Abnormal activation of the Wnt signaling pathway contributes to the occurrence and development of cervical cancer, colorectal cancer, and primary liver cancer. The Wnt signaling pathway is inhibited and regulated by many different antagonist molecules, such as sFRPs, WIF-1, and DKKs. In this study, we used DKK1 expression to reflect the status of the Wnt/*β*-catenin signaling pathway. We found that DKK1 was negatively expressed in most CSCs (64/116), and the DKK1 positivity rate was lower in patients with high clinical-stage, poorly differentiated tissues, deep muscle infiltration, or lymph node metastasis. After activation of the canonical Wnt/*β*-catenin signaling pathway, cytoplasmic *β*-catenin accumulates and enters the nucleus. Within the nucleus, *β*-catenin and TCF/LEF form a complex to initiate the transcription of Wnt target genes such as Snail1, Slug, and Twist, inhibiting E-cadherin expression and inducing EMT in a variety of tumor cells. We also performed expression validation. Of the 116 CSCs, 80 were positive for Twist2, of which 30 (37.5%) were positive for DKK1 expression. 36 cases were negative for Twist2, of which 22 (61.1%) were positive for DKK1 expression. The difference in expression of DKK1 and Twist2 was statistically significant (*P* < 0.05); DKK1 expression decreased with increasing Twist2 expression. We speculate that because DKK1 is an antagonist of the Wnt signaling pathway; reduced or absent DKK1 expression could cause abnormal activation of the Wnt signaling pathway and further upregulate Twist2 expression, thereby promoting EMT; this combination was also closely associated with the invasion and metastasis of CSC. Wnt family members regulate endothelial cell differentiation and vascular development and are associated with VM formation. In glioma and colon cancer tissues, the canonical Wnt/*β*-catenin pathway induces VM by promoting the expression of vascular endothelial growth factor receptor 2 (VEGFR-2) and VE-cadherin. However, there have been few related studies of CSC. To clarify the relationship between the expression of DKK1and VM formation in CSC, we evaluated DKK1, an important regulatory molecule of the Wnt/*β*-catenin pathway. The association of DKK1 with VM was analyzed by detecting DKK1 expression in CSC. DKK1 was detected in 50.6% (45/89) of the VM-negative group but 25.9% (7/27) of the VM-positive group. Furthermore, the OS analysis indicated that the patients who expressed DKK1 survived for more time than those who did not express DKK1. This difference was statistically significant, suggesting that DKK1 may be used as an indicator of CSC prognosis.

The article "Expression of Dickkopf-1 and Twist2 in Cervical Squamous Cell Carcinoma and Their Correlation with Vasculogenic Mimicry" was retracted in 2023. Reasons: signs of a paper mill; suspected computer-generated content; unreliable results or conclusions; concerns about the data.

## 5. Conclusions

This paper focuses on correlations among these factors as well as their correlation with clinicopathologic data and survival in CSC. DKK1, Twist2, and VM expression were immunohistochemically examined in 116 CSC tissues and 37 normal cervical tissues. The survival curve shows that the survival time of subjects with positive Twist2 and VM expression were lower than those with negative expression, the survival time with negative DKK1 expression was lower than positive expression; however, Cox multivariate analysis suggested that DKK1, Twist2, and VM were all independent factors for prognosis in patients with CSC, and therefore, we can speculate that the combined detection of DKK1, Twist2, and VM may be used as an indicator of CSC prognosis.

## Figures and Tables

**Figure 1:** Expression of DKK1, Twist2, and VM in CSC and normal cervical tissue. (a) Positive staining of DKK1 in CSC (400× magnification); (b) negative staining of VM in the control tissue (200× magnification); (c) positive staining of Twist2 in CSC (200× magnification); (d) negative staining of Twist2 in the control tissue (200× magnification); (e) positive staining of VM in the CSC (200× magnification); (f) negative staining of VM in the control tissue (200× magnification).

**Figure 2:** Kaplan–Meier analysis of the survival rate of patients with CSC. (a) Overall survival of all patients in relation to DKK1 expression; (b) overall survival of all patients in relation to Twist2; (c) overall survival of all patients in relation to VM.

**Table 1:** Expression of DKK1, Twist2, and VM in CSC and normal cervical tissues.

Clinical staging	Case number	DKK1 protein		*x* ^2^	*P* value	Twist2 protein		*x* ^2^	*P* value	VM expression		*x* ^2^	*P* value
−		+	−			+	−			+		
Normal cervix	37	12	25	5.8	0.016	23	14	11.473	0.001	37	0	10.46	0.001
Cervical cancer group	116	64	52			36	80		89	27		

**Table 2:** Relationships between DKK1, Twist2, and VM expression and clinicopathological parameters.

Clinicopathological parameters	Case number	DKK1		*P*	Twist2		*P*	VM		*P*
		−	+		−	+		−	+	
Age (years)										
<45	40	21	19	0.675	10	30	0.308	32	8	0.545
≧45	76	43	33		26	50		57	19	
Tumor diameter (cm)										
<4	51	24	27	0.12	15	36	0.738	40	11	0.700
≧4	65	40	25		21	44		49	16	
Clinical stage										
I	75	33	42	0.001	19	56	0.073	63	12	0.012
II	41	31	`10		17	24		26	15	
Pathological grade										
I(High)	31	9	22	0.003	13	18	0.042	27	4	0.005
II(Medium)	68	44	24		15	53		54	14	
III(low)	17	11	6		8	9		8	9	
With or without deep infiltration										
<1/2	47	20	27	0.024	20	27	0.027	41	6	0.027
≧1/2	69	44	25		16	53		48	21	
Lymph node metastasis										
−	81	37	44	0.002	31	50	0.010	68	13	0.005
+	35	27	8		5	30		21	14	

**Table 3:** Relationship between VM and DKK1.

Wnt/*β*-catenin-related protein	Total number	CSC		*x* ^2^	*P* value
		VM+	VM−		
DKK1					
+	52	7	45	5.08	0.024
−	64	20	44		

**Table 4:** Relationship between VM and Twist2.

EMT-related protein	Case number	CSC		*x* ^2^	*P* value
		VM+	VM−		
Twist2					
+	80	23	57	4.326	0.038
−	36	4	32		

**Table 5:** Relationship between DKK1 and Twist2.

Wnt/*β*-catenin-related protein	Case number	Twist2		*x* ^2^	*P* value
		+	−		
DKK1					
+	52	30	22	6.92	0.009
−	64	50	14		

**Table 6:** Results of univariate analyses of the overall survival (OS) time.

Clinicopathological parameters	Case number	5-year survival rate (%)	*x* ^2^	*P*
Age (years)				
<45	40	77.8	0.093	0.761
≧45	76	77.4		
Tumor diameter (cm)				
<4	51	81.7	0.974	0.324
≧4	65	74.1		
Clinical stage				
I	75	82.8	4.127	0.042
II	41	66.9		
Pathological grade				
I(High)	31	78.9	0.017	0.992
II(Medium)	68	77.2		
III(low)	17	75.1		
With or without deep infiltration				
<1/2	47	81.0	0.719	0.397
≧1/2	69	75.2		
Lymph node metastasis				
−	81	84.1	7.195	0.007
+	35	60.2		
DKK1 expression				
−	64	67.8	7.785	0.005
+	52	89.2		
Twist2 expression				
−	36	90.9	7.097	0.008
+	80	71.1		
VM expression				
−	89	83.4	10.382	0.001
+	27	53.9		

The article "Expression of Dickkopf-1 and Twist2 in Cervical Squamous Cell Carcinoma and Their Correlation with Vasculogenic Mimicry" was retracted in 2023. Reasons: signs of a paper mill; suspected computer-generated content; unreliable results or conclusions; concerns about the data.

**Table 7:** Cox multivariate analysis of the three factors and patient mortality.

Variable	*B*	SE	Wald	*P*	HR	95%CI
DKK1	0.995	0.474	4.408	0.036	2.704	1.068–6.846
Twist2	−1.228	0.623	3.883	0.049	0.293	0.086–0.994
VM	−1.068	0.413	6.668	0.010	0.344	0.153–0.773

## Data Availability

The datasets used and/or analyzed during the current study are available from the corresponding author on reasonable request.
